# Monitoring and Analysis of Youth Sports Physique by Intelligent Medical Robot Based on Cognitive Computing

This article has been retracted.

**DOI:** 10.1155/2022/5358059

**Published:** 2022-06-13

**Authors:** Yanming Pei, Yadong Chen

**Affiliations:** ^1^Sports Department, Shenyang Pharmaceutical University, Shenyang 110000, Liaoning, China; ^2^School of Physical Education, Shenyang Sport University, Shenyang 110032, Liaoning, China

## Abstract

As a key part of promoting the physical health of the people and promoting social progress, sports has ushered in comprehensive vitality. More and more people's attention has been paid to the physical health status, especially the physical status of young people. In the field of physical fitness monitoring, although the state has continuously increased investment in human and financial resources, it still cannot meet the needs of the market. This study mainly discusses the monitoring of youth sports physique by intelligent medical robots based on cognitive computing. This study introduces the development and implementation process of the management system and the test planning of the system. It focuses on the realization of the scalable architecture of the system server application and the communication mechanism of the intelligent terminal application. With the development of collaborative computing, social computing, and the ever-changing demands of human-computer interaction, it is difficult for a single user to take into account the interactive tasks in complex scenarios. The collaborative interaction of multiusers has gradually been paid more and more attention. Teenagers can log in to the intelligent medical robot system or mobile phone terminal to make health test appointments, score inquiries, and prescription inquiries. Its display module displays different contents according to different login identities. For teenagers, it is necessary to check personal physical test results and have a position on their physical health. Through the intelligent medical robot system, the administrator records and analyzes the results of the youth health test and gives appropriate exercise prescriptions for the youth. This not only analyzes the functional requirements that meet the basic user needs, but also analyzes the nonfunctional requirements that meet the most basic security, stability, and robustness of the software. Intelligent medical systems can effectively help people learn medical knowledge better in today's postepidemic era. It also helps people to conduct self-diagnosis and self-examination of minor diseases to a certain extent, so as to improve their own health. From the functional requirements, each module of the intelligent medical robot system is functionally described. From a nonfunctional point of view, the design and implementation meet the performance requirements of client-side robustness, maintainability, and stability. Finally, the system architecture of the intelligent medical robot is designed, and the specific database table is given. During the research, 20% of the students believed that their physical condition had been improved through physical health monitoring. The state of national physique can reflect a part of the country's comprehensive national strength to a certain extent. Throughout history, the overall development trend of a society and a country is constrained by the two factors of the group's constitution and economic development. This research will contribute to the physical and mental development of adolescents. The robot designed in this paper meets the requirements of a large number of students' centralized testing and is more accurate, faster, and more convenient.

## 1. Introduction

Adolescents are in the stage of growth and development, and their physical fitness is also in an important period of shaping. All kinds of sports quality can be further improved by scientific and reasonable development methods, and reasonable special physical fitness monitoring is beneficial to the improvement of special physical fitness. Therefore, the government needs to keep abreast of the dynamic changes of the national physical condition, especially the youth group. Based on the data obtained, it will be analyzed and the corresponding intervention measures will be taken. In addition, the physical fitness monitoring system is not only to evaluate the physical fitness level of athletes, but also to monitor the physical function changes of adolescents in real time. It can reasonably judge whether an athlete's training is scientific or not based on the changes in physical function of young people. Physical fitness is the foundation of study and work. Only with a good body can we work better to create value, realize the own ambitions, and realize the great Chinese dream.

In order to meet the requirements of centralized testing for a large number of students, more accurate, faster, and more convenient testing equipment is needed. It provides more reliable test equipment for relevant departments and units to carry out physical monitoring work and obtains accurate test data and results. Different kinds of fitness applications are aimed at users with different needs. However, with the development of fitness applications, they are becoming more and more homogenized, and more and more applications cover various types of functions, so as to expand the user group. The physical fitness monitoring system is not only to evaluate the physical fitness level of teenagers, but also to monitor the changes of physical function of teenagers. It can reasonably judge whether the training of teenagers is scientific according to the changes of the physical function of the athletes, so as to be beneficial to the improvement of the teenagers. Through the intelligent human-computer interaction interface, the workload of test staff is reduced, and the error caused by manual operation is reduced at the same time. It can realize multiperson and multimachine testing at the same time through wireless communication, saving time and staff.

Simultaneous testing can accommodate long-distance transmission (e.g., playgrounds, gymnasiums). Each device is relatively independent for easy installation and transportation. The equipment adopts a highly integrated design, which makes each equipment easy to install. It firstly obtained the data of physical health monitoring of adolescents and extracted some adolescents' physical fitness monitoring data to analyze the average, standard deviation, and correlation coefficient of the group of adolescents' body shape and motor function. The purpose is to understand whether the sample obeys the normal distribution and to find out the current situation of adolescents' physical health through descriptive statistics. It uses wireless connection to collect data from multiple devices, which makes the connection between computers and devices very convenient. Most of the current cognitive computing research is based on the analysis of single-channel data, such as cognitive computing based on EEG data, cognitive computing based on eye movement data, etc. However, whether it is eye movement data or EEG data, all that can be obtained is a part of the information related to the user's cognition. It is mainly designed around projects such as sit-ups, pull-ups, and skipping ropes. It simultaneously measures the acute and long-term effects caused by the test of these physical indicators and observes the relationship and development ratio between related indicators such as body shape, function, and biochemistry. It is used as an evaluation of physiological and biochemical effects in addition to training evaluation.

## 2. Related Work

The intelligent mobile terminal of the intelligent medical robot system has been widely used in a variety of traditional industries. Its flexible operation, user-friendly user experience, rich functions, and free open source code make it very popular among users and manufacturers in various fields. The national physique comprehensive evaluation model only needs to analyze the feature importance of the national physique comprehensive evaluation model by correlating the personal physique test information and find the root node in combination with the information gain. Hayat S believes that, in recent decades, the use of antibody drug conjugates (ADCs) has brought hope for the treatment of cancer. This smart drug delivery system is also named Armed Antibody. He describes important factors in ADC design and performance. He searched Pubmed, Scopus, Web of Science, and other databases with “Antibody Drug Conjugate” as the keyword and screened out 58 related articles published from national physique comprehensive evaluation from 2000 to 2017. To develop a suitable ADC, different parameters should be considered. The selection of antibody, drug, and linker types should be based on different factors to achieve ADCs with optimal performance. To date, more than 671 clinical trials have been registered in the Clinical Trials Database Registry using the keyword “antibody drug conjugates”. But only three drugs under the trade names Mylotarg, Adcetris, and Kadcyla have been approved by the FDA, and production of Mylotarg was halted due to lethal effects. Traditional methods of treating cancer have adverse effects due to the effects of chemotherapeutic drugs on normal cells, but the use of ADCs can induce tumor cell apoptosis through targeted drug delivery [1]. Bo T believes that data-intensive analytics is a major challenge for smart cities due to the ubiquitous deployment of various sensors. The natural characteristics of geographic distribution require a new computing paradigm to provide location-aware and latency-sensitive monitoring and intelligent control. His fog computing, which extends computing to the edge of the network, meets just that need. He introduced a layered distributed fog computing architecture to support the integration of numerous infrastructure components and services in future smart cities. To protect future communities, it is necessary to integrate intelligence into fog computing architectures. For example, it performs data representation and feature extraction, identifies abnormal and hazardous events, and provides optimal response and control. He analyzes case studies using an intelligent pipeline monitoring system based on fiber optic sensors and sequential learning algorithms to detect events that threaten pipeline safety [2]. Karlowsky et al. use the microdilution method used in the laboratory standard study. This determined the in vitro susceptibility of a Gram-negative ESKAPE pathogen machine isolated from hospitalized patients with intra-abdominal infection (IAI) (*n* = 3052) and urinary tract infection (UTI) to eight parenteral antimicrobials [3]. Chen et al. believe that the gap between computational and semantic features is one of the main factors hindering the performance of computer-aided diagnosis (CAD) for clinical use. To bridge this gap, they use deep learning models derived from Stacked Denoising Autoencoders (SDAE) and Convolutional Neural Networks (CNN), as well as handcrafted Haar-like heterogeneous computational features and HoG features. This is used to describe 9 semantic features of lung nodules in CT images. They believe that there may be relationships between semantic features such as “spiculation, texture, and margin,” which can be explored with MTL. They use the Lung Image Database Consortium (LIDC) data for a rich source of annotation. By treating each semantic feature as a separate task, the MTL scheme evaluates selection and maps heterogeneous computational features to radiologists' scores through cross-validation [4]. Muhammad et al. believe that the integration of IoT and cloud technologies is important to provide better solutions for uninterrupted, secure, seamless, and ubiquitous frameworks. The complementarity and capabilities of IoT in storage, processing, accessibility, security, service sharing, and components make convergence suitable for many applications. Advances in mobile technology have added a degree of flexibility to this solution. The health industry is one of the places that can benefit from IoT-cloud technology due to factors such as scarcity of professional doctors and physical activity limitations of patients. As a case study, they discuss the feasibility of using IoT-cloud to monitor speech pathology in people and propose a solution [5]. In terms of hardware, an independent upper computer and lower computer are designed. The independence of the equipment is convenient for installation, transportation, and use, which solves the cumbersome wiring and debugging links of traditional equipment. At the same time, the interface of traditional hardware equipment is expanded, which is convenient for existing enterprises to reduce costs. The main purposes of the standardization of national physique monitoring data include the following: Through the standardization of the data storage format, after the administrator uploads the physical fitness test data, the database of the service application platform can reduce errors and improve the work efficiency of the administrator after receiving and processing the physical fitness test data. On the other hand, it can also lay a solid foundation for the establishment of a comprehensive evaluation model of national physique and a fitness mode recommendation model and complete the development of a service application platform. The intelligent physique monitoring system designed this time is completed under the condition of combining the new concept of youth physique health status and intelligent Internet in the new era. The system is designed and implemented according to the original design scheme and completed according to the predetermined plan, and some functions are improved and expanded.

## 3. Monitoring and Analysis of Youth Sports Physique by Intelligent Medical Robot Based on Cognitive Computing

### 3.1. Structural Layer Design of the Robot System for Adolescent Physique Monitoring and Health Assessment

#### 3.1.1. The Presentation Layer of the National Physique Monitoring and Health Assessment Robot System

It mainly refers to the main platform for the interaction between the robot system and the user, that is, the front-end page display part of the juvenile physique monitoring and health assessment robot system. In the adolescent physique monitoring and health assessment robot system, the presentation layer mainly realizes a reasonable and easy-to-use web interface through HTML, CSS, JavaScript, and other front-end language design. It presents the data required by the robot system to the user reasonably and completely. At the same time, the layout of the controls in the web page is reasonably arranged, so that the user can interact with the robot system very conveniently. In addition, the presentation layer of the youth physique monitoring and health assessment robot system can also monitor the events triggered by the user in real time and accept the user's request. It makes different judgments according to different requests of users and sends the requests. In the adolescent physique monitoring and health assessment robot system, there is only interaction between the business logic layer and the presentation layer. In addition, the page caching technology provided by ASP.NET is also used in the presentation layer of the juvenile physique monitoring and health assessment robot system. When users frequently make similar requests, the page cache server will directly fetch the results from the cache. This reduces the number of times the robot system frequently processes similar requests and improves the operation efficiency of the robot system. However, generating dynamic web pages consumes enormous resources. Every change in the page needs to send a request from the browser to the server, and then the server extracts the relevant information from the database. And its connection to the database also requires additional consumption of limited connection resources to access the database (the youth physical fitness monitoring and health assessment robot system uses a database connection pool). However, obtaining these resources also requires resource competition or waiting, resulting in more resource overhead. In addition, due to the frequent access to the data by the adolescent physical fitness monitoring and health assessment robot system, it is necessary to use page caching technology for pages with relatively small changes.

The specific probability is expressed as [6]

(1) $$\begin{array}{c} P\left(X=K\right)=C_{m}^{k}*{\left(\frac{1}{T}\right)}^{K}*{\left(1-\frac{1}{T}\right)}^{m-k}. \end{array}$$

The probability that only one label is selected for a slot is [7]

(2) $$\begin{array}{c} P_{G}=P\left(X=1\right)=C_{m}^{1}*\left(\frac{1}{T}\right)*{\left(1-\frac{1}{T}\right)}^{m-1}=\frac{m}{T}*{\left(1-\frac{1}{T}\right)}^{m-1}. \end{array}$$

When *k*=0 [8]:

(3) $$\begin{array}{c} P_{l}=P\left(X=0\right)=C_{m}^{0}*{\left(\frac{1}{T}\right)}^{0}*{\left(1-\frac{1}{T}\right)}^{m-0}={\left(1-\frac{1}{T}\right)}^{m-1}. \end{array}$$

Then when *k* ≥ 2, the probability of collision time slot [9]:

(4) $$\begin{array}{c} P_{G}=P\left(X\geq 2\right)=1-P\left(X=1\right)-P\left(X=0\right). \end{array}$$

The specified system throughput rate *S*_*R*_ is

(5) $$\begin{array}{c} S_{R}=\frac{a}{T}=\frac{m}{T}{\left(1-\frac{1}{T}\right)}^{m-1}. \end{array}$$

Its derivation can be obtained [10]:

(6) $$\begin{array}{c} \frac{\text{d}s}{\text{d}m}=\frac{1}{T}{\left(1-\frac{1}{T}\right)}^{m-1}+\frac{m}{T}{\left(1-\frac{1}{T}\right)}^{m-1}\ln\left(1-\frac{1}{T}\right). \end{array}$$

#### 3.1.2. The Business Logic Layer of the Youth Physique Monitoring and Health Assessment Robot System

The core part of the robot system for juvenile physique monitoring and health assessment is the business logic layer of the robot system. The request processing and operations between the user and the adolescent physical fitness monitoring and health assessment robot system all need to be processed by the business logic layer. The business logic layer is the bridge connecting the presentation layer and the data layer. The main purpose of the three-tier architecture of the B/S model is to realize the decoupling of the software robot system. Through the processing of the business logic layer, the presentation layer only needs to call the interface provided by the business logic layer to complete the relevant work. The data layer only needs to wait for the notification after the business logic layer completes the data processing and is in a passive calling state. Therefore, modifying the function of the presentation layer will not affect the realization of the business logic layer, and the modification of the business logic layer will not affect the database to complete its own work. The existence of the business logic layer is the key to support the scalable architecture of the youth physique monitoring and health assessment robot system. The business logic layer plays the role of connection and communication in the middle of the two layers. It plays two different roles of calling and being called. From the perspective of the business logic layer, it is not only the caller of the data layer, but also called by the presentation layer. The relationship between dependencies and dependents is well represented in the business logic layer. Therefore, in order to ensure the decoupling of the design of the youth physique monitoring and health assessment robot system and realize the complete separation of the development process of the robot system, we designed the business logic layer as an alternative and extractable drawer architecture.

#### 3.1.3. The Data Layer of the Youth Physical Fitness Monitoring and Health Assessment Robot System

The data layer is also called the data persistence layer, which implements the data persistence logic. It is mainly responsible for the data saving and reading functions in the youth physical fitness monitoring and health assessment robot system. It has nothing to do with the business logic of the adolescent physique monitoring and health assessment robot system. Because the ASP.NET development platform is used in the juvenile physique monitoring and health assessment robot system, the data persistence layer of this robot system is mainly realized through ADO.NET. ADO.NET comes from the COM component library ADO (ActiveXDataObjects). It is currently the main interface for developing NET database applications. It is the access model of the new generation of Microsoft's NET database. It uses NETDataProvider (data provider) for database access and connection. It can use a variety of objects to access database content in ADO.NET database programs. This enables various manufacturers of database management robot systems to open the corresponding NETDataProvider according to this standard. This allows developers who design database applications to access any database that supports NETDataProvider only through the object model provided by ADO.NET, without knowing the underlying operational details of the database. Therefore, we use ADO.NET to access the data in a robotic system for adolescent fitness monitoring and health assessment. Through the analysis of the three-tier architecture of the B/S model, it can be clearly understood that the three-tier architecture meets the low coupling requirements of the youth physique monitoring and health assessment robot system. This makes maintenance of the entire robotic system much easier. The business logic layer of the robot system uses the access interface provided in the data layer to access the data in the database. On the browser side, the youth physique monitoring and health assessment robot system calls the interface provided by the business logic layer through the browser interface.

The functional relationship between the number of time slots and the number of tags can be obtained by finding the extreme value as [11]

(7) $$\begin{array}{c} T=\frac{1}{1-e^{-1/m}}\approx m+1. \end{array}$$

It uniformly maps the data to the [0, 1] interval, and its transformation function is [12]

(8) $$\begin{array}{c} X^{\prime }=\frac{X-X_{\min}}{X_{\max}-X_{\min}}. \end{array}$$

*X*_min_ is the minimum value of the data in the dataset; *X*_max_ is the maximum value of the data in the dataset.

The Pearson correlation coefficient *ρ* for variables *x* and *y* is [13]

(9) $$\begin{array}{c} \rho =\frac{\sum \left(x-\bar{x}\right)\left(y-\bar{y}\right)}{\sqrt{\sum \left(x-\bar{x}\right)\sum \left(y-\bar{y}\right)}}. \end{array}$$

The mutual information of *x* and *y* defines *I* as [14]

(10) $$\begin{array}{c} I=\sum \sum_{\text{i}=1}p\left(x,y\right)\log\frac{p\left(x,y\right)}{p\left(x\right)p\left(y\right)}. \end{array}$$

The maximum correlation and minimum redundancy are calculated as [15]

(11) $$\begin{array}{c} \max D_{S}=\frac{1}{{\left|S\right|}^{2}}\sum I\left(X,C\right),\\ \max R_{S}=\frac{1}{{\left|S\right|}^{2}}\sum I\left(X_{i},X_{j}\right). \end{array}$$

### 3.2. Functional Design of Robot System

This robot system mainly provides different health advice for people and improves people's quality of life by monitoring the physical fitness of different groups of people of all social strata and age groups. Users of this robot system can log in to their respective accounts to view their own physical fitness monitoring results and can view statistical charts of their own physical fitness changes over a period of time, allowing users to more easily understand their own physical fitness changes. The robot system can also give corresponding health improvement plans according to the assessment results of individual physique. Users can further strengthen their physical fitness and reduce the risk of disease according to the plan. In addition, the robot system administrator can also perform statistical analysis on the health status of groups in relevant regions or age groups, providing the basis for research and analysis for relevant organizations. The design of the functional modules of the robot system is shown in Figure 1.

#### 3.2.1. User Management Module

This module consists of two parts, one is the administrator user, and the other is the ordinary user. Ordinary visitors can become ordinary users of the website by registering on this website. After logging in to the robot system, ordinary users can browse the basic information of their own accounts and modify some of their own information. The administrator user logs in with the user account provided by the company. Administrator users can also modify some basic information of their own account. In addition, administrator users can also query the basic information of ordinary users and enter the physical examination results of ordinary users. The user management module includes three functions: user login, user registration, and personal information management. In the juvenile physique monitoring and health assessment robot system, the user first needs to verify the identity through the login operation. Only after the identity verification is successful can they view their personal basic information and physical fitness monitoring results and other information.

#### 3.2.2. Physical Fitness Monitoring Module

In the physical fitness monitoring module, users can upload their physical examination information to the robot system by themselves or through the administrator. The robot system will automatically evaluate the user's health status based on the information uploaded by the user and display the evaluation results on the website. Users can also understand the changes in their physical health over a period of time by viewing historical information. When users need to perform physical fitness monitoring, they can log in to the adolescent physical fitness monitoring and health assessment robot system in advance to make an appointment. After the appointment is successful, they go to the physical monitoring institution for physical monitoring. The monitoring results will be automatically displayed in the user's personal health information, and the user can query it after logging in to the adolescent physique monitoring and health assessment robot system.

#### 3.2.3. Statistics Reporting Module

In the statistical reporting module, a variety of statistical analysis methods are provided for the robot system administrator. The youth physique monitoring health assessment robot system can divide the user's physical health status from different age groups. This allows relevant personnel to better analyze the health status of different age groups. It divides the user's health status from different health indicators to understand which groups of subhealth status are mainly concentrated and so on. This is the need for relevant institutions to conduct further overall analysis on the physical condition of adolescents. In addition, a data reporting function is designed for the adolescent physique monitoring and health assessment robot system. The robot system administrator can report relevant data information and overall analysis results to the physical fitness monitoring center.

#### 3.2.4. Robot System Management Module

The youth physique monitoring and health assessment robot system management module can make it more convenient for administrators to manage various data information in the robot system and improve the business logic. In the robot system management module, after logging in to the robot system, the administrator user can perform related management and batch addition operations to the users registered in the robot system. For the user's physique monitoring appointment information, the robot system administrator can manage the overall management and query the detailed appointment information of individual users or the appointment status of related institutions. The management of monitoring agencies also belongs to the category of robot system management. Administrators can add new physical fitness monitoring institutions, modify outdated monitoring institution information, and conduct overall management of monitoring institutions.

#### 3.2.5. Health Promotion Module

The youth physique monitoring and scientific fitness guidance module designed and implemented by this research group is a closed-loop health promotion service module. It includes five links: physical fitness testing, health assessment, exercise prescription, exercise intervention, and tracking feedback. It provides adolescents with integrated services ranging from data collection, health assessment, and prescribing interventions to follow-up feedback. Among them, the physical fitness test is to obtain and save the youth physical fitness data and motor function data through a series of health physical fitness testing equipment and intelligent fitness equipment. Health assessment is a comprehensive assessment of the health status of adolescents based on adolescent health signs data, motor function data, and questionnaire results. It identifies the health risks faced by adolescents and locks adolescents' health management goals and healthy cardiovascular risk stratification levels. Exercise prescription is to formulate an effective exercise prescription based on the comprehensive evaluation of adolescents' physical exercise data and health management goals. Exercise intervention means that, after getting a scientific exercise prescription, teenagers exercise according to the prescription instructions and evaluate their motor feelings after the exercise. Tracking feedback is to continuously adjust exercise intensity, exercise time, and exercise energy consumption settings according to the result feedback during the process of adolescents' implementation of prescriptions, so as to ensure that adolescents implement correct exercise programs. The program setting of the health promotion module is shown in Figure 2.

### 3.3. Physical Fitness Detection Submodule

The physical fitness submodule is used to display user management goals and physical fitness data. It mainly consists of three parts of data: the management target part, the health physical test part, and the exercise ability test part. The management goals section mainly displays the user's management goals and cardiovascular risk stratification levels. Management target results and cardiovascular risk stratification levels are obtained by analyzing user questionnaires and other physical examination data through the cloud service platform. Users can click the management target to enter the secondary menu to view the user health report. The health fitness test section displays the latest test results of the health fitness index data. It includes the indicator name and indicator value and is not displayed without testing. The sports ability test part displays the latest test results of sports items, including the names and values of various indicators.

It first constructs the loss function [16]:

(12) $$\begin{array}{c} J=\frac{1}{N}{\sum \left(f\left(x\right)-y\right)}^{2}=\frac{1}{n}{\sum \left(wx-y+b\right)}^{2}. \end{array}$$

The solution form of *w* is

(13) $$\begin{array}{c} w=\arg\min{\left(y-Xw\right)}^{T}\left(y-Xw\right). \end{array}$$

The final solution *w* can be obtained by derivation [17]:

(14) $$\begin{array}{c} J=\frac{1}{N}{\sum \left(F\left(X\right)-Y\right)}^{2}+\chi \left\|W\right\|. \end{array}$$

Ridge regression adds regularization term *L*_2_ to the loss function, and its specific formula is [18]

(15) $$\begin{array}{c} W={\left(X^{T}X+\lambda I\right)}^{-1}X^{T}Y. \end{array}$$

The SVM regression problem can be formalized as [19]

(16) $$\begin{array}{c} R_{M}=\text{MIN}{\left\|w\right\|}^{2}+c\sum I\left(f\left(x\right)-y\right). \end{array}$$

### 3.4. Motion Module Implements

It is used to request exercise prescriptions and monitor the execution of both custom and prescription exercises. Users can apply for a prescription after meeting the prescription application conditions. The cloud service platform analyzes the user's prescription according to the user's data and sends the prescription to the client after the user's request. Today's prescription is a list of the most recently requested prescription exercises by the user. Prescription exercises indicate exercise type, energy consumption, duration, and completion status, and some prescription exercises have skip signs. Today's prescription interface is implemented by UIScrollView. Each row is a UIView, instantiated and added to the UIScrollView. There are three main types of prescribed exercise: warm-up, endurance, and finishing. Exercise energy consumption and exercise time settings are determined according to the user's physical data. Prescription exercise completion status includes completed, incomplete, and skipped. It will change according to the user's specific exercise situation, and for prescriptions that are not marked with skip signs, the user can only execute them sequentially. After the prescription exercise, it uploads the prescription exercise result data to the cloud service platform as the basic data for the next analysis. Custom sports mainly list some regular sports, such as cycling, running, walking, swimming, etc. These movements are presented in the form of a table, each row shows three movements, and the specific number of rows is determined according to the result returned by the server. For each sport, the client will display the sport's image representation, name, and sport evaluation. Motion evaluation is performed at the same time as the user motion is completed and submitted. If the user does not comment, the result of this exercise cannot be submitted. The user reservation table saves the information of the current reservation user. The specific information when the user makes an appointment is shown in Table 1.

In the user information table, the basic information of the user is mainly stored. Due to the privacy of the physical fitness monitoring information, in order to ensure the information security of each user, the user needs to register on this website and log in correctly before viewing the basic information of the user. After users enter their username and password, they can click to log in. The system first goes back to visit the user information table in the database, compares the information entered by the user with the data in the user information table, and allows the user to use the system functions after the comparison is successful. The specific data of user information are shown in Table 2.

### 3.5. Mobile Terminals

The mobile terminal is a part of the youth physique monitoring and scientific fitness guidance system. It is an innovative part and also the research topic of this paper. It directly interacts with users, collects data on users' personal physique, exercise, etc., monitors users' prescription movements, and conducts data interaction with the cloud through the network. Therefore, from a small scope, it includes three modules: cloud storage, cloud service, and mobile terminal. Among them, the cloud storage uses MySQL to store data, including physical fitness monitoring data, questionnaire survey result data, exercise monitoring data, and heart rate data. The cloud service module uses data mining technology to analyze and reason the data in the cloud storage module. It gets the scientific exercise prescription and saves it to the cloud storage module. The mobile terminal indirectly interacts with the MySQL database of the cloud storage module through the cloud service. This method can realize the distributed data processing, reduce the coupling between the mobile terminal and the remote database operation, and increase the cross-platform operability. The trend of youth physique data is shown in Figure 3.

It introduces slack variable *ϑ*:

(17) $$\begin{array}{c} R_{M_{\vartheta }}=\text{MIN}{\left\|w_{\vartheta }\right\|}^{2}+c\sum I\left(f\left(x\right)-y_{\vartheta }\right). \end{array}$$

The Lagrangian function can be obtained by introducing the Lagrangian multiplier [20]:

(18) $$\begin{array}{c} f\left(x\right)=\sum \left(\varphi -\varphi_{i}\right)l\left(x,x_{i}\right)+b. \end{array}$$

The designed fitness function:

(19) $$\begin{array}{c} f\left(x\right)=\beta R\left(x\right)+\left(1-\beta \right)\left(1-\frac{n}{N}\right). \end{array}$$

*n* represents the number of currently selected features.

The designed crossover probability *P*_*J*_ and mutation probability *P*_*b*_ are [21]

(20) $$\begin{array}{c} P_{J}=\left(1-\frac{g}{G}\right)\phi \frac{f_{\max}-f}{f_{\max}-f_{\text{avg}}},\\ P_{\text{b}}=\left(1-\frac{g}{G}\right)\theta \frac{f_{\max}-f}{f_{\max}-f_{\text{avg}}}. \end{array}$$

The mathematical expression for the hyperparameter optimization problem is

(21) $$\begin{array}{c} X=\arg\min S\left(X\right). \end{array}$$

Gaussian process formula [22]:

(22) $$\begin{array}{c} f\left(x\right)=GP\left(m\left(x\right),k\left(x,x^{\prime }\right)\right). \end{array}$$

*k* in the formula is the covariance function, and this paper uses the exponential square function as the covariance function [23]:

(23) $$\begin{array}{c} k\left(x,x_{i}\right)=\exp\left(1-\frac{1}{2}{\left\|x_{i}-x_{j}\right\|}^{2}\right). \end{array}$$

## 4. Monitoring Results of Youth Sports Physique

In 2017, the proportion of the number of adolescents whose physique reached the “qualified” standard for adolescent physique increased by 0.7 percentage points. There is an increasing trend for different age groups, different genders, and urban and rural populations, especially in rural and female populations. This in turn reflects an overall improvement in youth fitness levels 22. However, there are also unbalanced developments. The physiques of adolescents in different regions are shown in Table 3.

After the physical fitness monitoring is completed, the user submits the monitoring results to the physical fitness monitoring health assessment system. The system will compare the monitoring results with the national physique measurement standards to obtain corresponding scores. For the height, some scoring standards of the physical fitness measurement items are shown in Table 4.

The juvenile physique monitoring robot will regularly send juvenile physique reports. The physique report sheet of adolescents is shown in Figure 4 [24–26].

In the reaction layer, the evaluation results of the five indicators are mostly good, and the proportions are higher than other grades. This shows that students still agree with their cognition and attitude towards physical health monitoring. In the second indicator of the reaction layer, “the motivation to participate in physical fitness monitoring is clear”, choose a medium proportion, and the purpose of participating in physical fitness monitoring is to correctly understand the significance and function of physical fitness monitoring. It can be seen that most students do not have a clear understanding of the motivation of physical health monitoring. This may be because the publicity of physical fitness monitoring is not enough, and it has not been paid much attention by teachers and classmates, so the understanding of motivation is not particularly clear. In the overall evaluation analysis of the reaction layer, excellent evaluation accounted for 29.6%, good evaluation accounted for 42.5%, moderate evaluation accounted for 24.7%, low evaluation accounted for 3.2%, and the overall score was 84.88 points; the evaluation was good. The evaluation of the reaction layer results is shown in Figure 5.

In the results of the behavior level, most of the students expressed their willingness to insist on participating in activities such as physical fitness monitoring, and the excellent and good rate reached 75%. Nearly 70% of the students expressed their willingness to insist on participating in physical exercise, accounting for the majority of the evaluation grades. When it comes to whether they can do physical exercise correctly, 14% of the students are at a low level, so the guidance on physical exercise should be strengthened. But in general, the students in this class have achieved excellent changes in physical exercise behavior through participating in physical fitness monitoring. According to the overall evaluation analysis of the behavior level, excellent evaluation accounted for 19.6%, good evaluation accounted for 45.7%, medium evaluation accounted for 28.2%, and poor evaluation accounted for 6.6%. The overall score is 82.91 points, which is rated as good. The evaluation results of the behavioral layer analysis are shown in Figure 6.

In the seven evaluation indicators of the learning layer, the proportion of excellent grades is mostly. It can be seen that, through this physical fitness monitoring, the students in this class have learned a certain amount of knowledge and have a good grasp of the test content. In the motor skills of the test items, the proportion of selected and so on is also more than other evaluation grades. The reason may be that the mastery of motor skills is largely determined by the students' physical quality and skill level, thus affecting their mastery. There is an indicator for the level of poor evaluation, which is the evaluation method of the test content. The reason for the analysis may be that there are differences in the test data on the same item, which leads to the ambiguity of students' evaluation methods. But overall, the evaluation results of the learning layer are still good [27, 28]. In the overall evaluation analysis of the learning layer, the excellent evaluation accounted for 28.2%, the good evaluation accounted for 42.3%, the medium evaluation accounted for 23.7%, and the poor evaluation accounted for 5.8%. The overall score is 84.24 points, which is rated as good. The results of the learning layer analysis are shown in Figure 7.

In the result layer, 18%, 24%, and 20% of the students, respectively, believed that physical health monitoring enhanced their awareness of maintaining healthy exercise, developed good physical exercise habits, and improved their physical condition, and they expressed their strong agreement, which is an excellent level. In the three indicators of the result layer, the proportions in the good level are 55%, 39%, and 39%, respectively. In the overall evaluation analysis of the result level, excellent evaluation accounted for 20.2%, good evaluation accounted for 44%, medium evaluation accounted for 21.4%, and poor evaluation accounted for 7.5%. The overall score was 77.52 points, and the evaluation was moderate. The result layer analysis is shown in Figure 8.

In order to better store and access user information, it is necessary to create a reasonable database table for the project to realize the operation of various user information. The database used in the project is MySQL, which is a widely used relational database. Database tables are designed in a top-down fashion. After analyzing the overall requirements of the system, the database tables required by each module are refined step by step, so as to reduce the connection between the tables. The performance evaluation design is shown in Table 5.

Through this system, the students' test summary scores are generated, and the overall analysis and description of the students' comprehensive scores are carried out. Taking the boys from the first class of 2017 as the subjects of the intervention, we can clearly see that three of them failed. The summary results of the health test are shown in Table 6.

The overall compliance rate of middle school students' physical health status is mainly distributed in two grades: pass and good. The excellent rate is 1.55%, the good rate is 23.87%, and the pass rate is 92.24%. The overall compliance rate of middle school students' physical health status is shown in Figure 9.

## 5. Discussion

The key to a computer's ability to generate insight is to enable it to interpret unstructured data, and the key to this technology is cognitive computing. By designing an algorithm system, the computer simulates the way of human thinking and realizes the interpretation of unstructured data. It is also for this reason that cognitive computing is considered a necessary technology for the future data generation.

Robotics is one of the most comprehensive and attractive application fields of artificial intelligence research. In the past half a century, it has been developed by leaps and bounds, and its application range covers industry, agriculture, civil, military, and other aspects, for example, from painting and assembly robots that replace human mechanical operations on industrial production lines, to intelligent mobile robots, to lunar rovers and Mars rovers. At present, the more mature and successfully applied robots are mainly in specific environments and for specific tasks. With the continuous improvement of the demand for intelligence level, human beings increasingly need human-like intelligent robots that can work in a highly complex environment, perform nonspecific tasks, and have a high degree of autonomy.

For the exchange and sharing of physical fitness test data, the service application platform (referring to the national physical fitness monitoring system and other fitness systems that store physical fitness test data) will automatically generate an open format definition file according to the basic rules of physical fitness test data exchange. It includes the location of physical fitness test data storage, the name of the data table, the data structure of the system, etc., to realize the establishment of data files. This thus stores the shared data files and information, etc. in the intermediate database. The visual learning method based on the cognitive computing model of the human brain possesses some of the above cognitive abilities. This enables the vision system based on this model to deal with the problems that cannot be solved by the traditional vision system and constantly adapt to the complex and uncertain environment, and the level of intelligence is greatly improved.

Based on the background of cognitive computing, machine learning is used to mine the value of historical data of physical fitness test and complete the development of service application platform. This not only has a certain significance for the informatization development of the national physique monitoring work, but also can promote the national physique monitoring management and research work to gradually move towards a higher stage of informatization and at the same time further promote the intelligent construction of mass sports. This research can not only realize automatic data processing for the national physique monitoring system, fitness platform, etc., but also provide a preset scheme of data standardization. It can also provide a reference method for data mining of physical fitness test and fitness method recommendation algorithm. At the same time, the development of its service application platform can also contribute to improving the timeliness, efficiency, and scientificity of the collection, processing, and analysis of national physique monitoring data.

In the national physical fitness monitoring work, after each related work is completed, the staff will collect and organize all physical fitness test data. They store the processed data in the physical fitness test server of the country or the corresponding province and city. However, as far as managers are concerned, there are still some problems in the efficiency of data processing. Real-time viewing of physical fitness test details in each district needs to be improved. As far as physical fitness testers are concerned, there is a need to modify and view basic information such as personal physical fitness tests. In addition, for nonprofessionals, they may not know much about the national physique monitoring work and related professional terms, and the specific meaning of the data is not clear.

At present, the national physical fitness monitoring work in China is relatively mature, and a large amount of historical data of physical fitness testing has been accumulated. In addition, in the information age, big data has gradually attracted the attention of scholars in the monitoring of national physique. Data hides infinite value, and the development of machine learning is to add bricks and mortar to the technology of mining the value of data. In general, for the relevant research on the national physique monitoring, the country should not only pay attention to the development of the physique monitoring work, but also pay more attention to the standardization of the national physique monitoring data. It should also focus on using the combination of machine learning and data mining technology to activate the historical data of physical fitness test and mine the value of data. It provides a preset scheme to promote the sharing and exchange of physical fitness monitoring data.

## 6. Conclusion

Today, with the rapid development of smart hardware, more and more new technologies have been proposed, and more and more manufacturers have joined this wave, especially smart wearable devices. Now health, physique, and exercise have become social hotspots. From the country, the organization, to the ordinary people, they are more and more concerned about the physical health of themselves and the next generation. As another process of realizing the core business of this system, the health intervention function is also the core of developing this system. By analyzing the performance of the teenagers, the administrator puts forward suggestions on healthy exercise for the teenagers. After the suggestion is generated, the system will send a suggestion content message to the designated teenagers. After receiving the message, teenagers can log in to the system to view the healthy exercise suggestions given by teachers. It should be seen that the college students' health test management system is a part of sports network teaching. Although there has been obvious improvement in the effect of physical education and the enthusiasm of students, it also has some limitations. It cannot completely replace the traditional face-to-face physical health consultation education, but only supplement the traditional teaching. With the continuous development and improvement of network, multimedia and other technologies, traditional physical education and network teaching will be better combined, and the network teaching platform of physical education will become more and more perfect.

## Figures and Tables

**Figure 1:** Design of functional modules of robot system.

**Figure 2:** Scheme setting of the health promotion module.

**Figure 3:** Trends in youth physique data.

**Figure 4:** Adolescent's physical fitness report.

**Figure 5:** Evaluation of the reaction layer results.

**Figure 6:** Evaluation of analysis results at the behavioral level.

**Figure 7:** Learning layer analysis results.

**Figure 8:** Results layer analysis.

**Figure 9:** The overall compliance rate of middle school students' physical health status.

**Table 1:** Specific information when users make an appointment.

Serial number	Field name	Length	Is it empty
1	Appointment id	11	No
2	Appointment user	11	No
3	Appointment company	11	No
4	Appointment date	4	No
5	Appointment_ height	4	Yes

**Table 2:** Specific data of user information.

Serial number	Field name	Type of data	Length
1	User_id	Int	11
2	User_login	Varchar	20
3	User_password	Varchar	8
4	User_name	Varchar	20
5	User_sex	Varchar	20

**Table 3:** Adolescent physique in different regions.

Province (region, city)	Overall	Town	Rural	Male	Female
1	91.6	95.5	84.5	90.1	93.0
2	91.7	93.8	88.3	91.4	92.0
3	93.0	94.2	91.3	93.1	92.9
4	84.1	86.9	79.6	81.9	86.4
5	93.0	96.9	86.3	91.5	94.4

**Table 4:** Partial scoring criteria for physical fitness measurement items for height.

Height	1 point	2 points	3 points
170.0–170.9	<52.0	52.0–55.7	55.8–72.1
171.0–171.9	<52.7	52.7–56.6	56.7–73.1
172.0–172.9	<53.5	53.5–57.5	57.6–74.0
173.0–173.9	<54.1	54.1–58.3	58.4–75.0

**Table 5:** Performance assessment design.

Number	Column name	Type of data	Describe
1	Grade_id	Int	User grade id
2	User_id result	Float	Fraction
3	Is_ reach	Int	Is it up to standard
4	Rank	Int	Ranking

**Table 6:** Health test summary scores.

Serial number	Endurance class results	Flexibility and strength	Speed and dexterity category	Overall grade
1	59	−0.4	2.29	Pass
2	48	8.7	2.17	Pass
3	47	−2.8	1.77	Failed
4	59	6.8	2.19	Failed
5	47	8	2.06	Pass
6	55	3.8	2.56	Failed

## Data Availability

No data were used to support this study.
